The article "Deep Learning Algorithm-Based Ultrasound Image Information in Diagnosis and Treatment of Pernicious Placenta Previa" was published in 2022. Journal: Comput Math Methods Med.

# Deep Learning Algorithm-Based Ultrasound Image Information in Diagnosis and Treatment of Pernicious Placenta Previa

**DOI:** 10.1155/2022/3452176

**Published:** 2022-06-06

**Authors:** Xiao Yang, Zheng Chen, Xiaozhou Jia

**Affiliations:** ^1^Department of Obstetrics and Gynecology, Hunan Provincial Maternal and Child Health Care Hospital, Changsha, 410008 Hunan, China; ^2^Department of General Surgery, The First Hospital of Changsha, Changsha, 410005 Hunan, China

## Abstract

This study was to explore the value of the deep dictionary learning algorithm in constructing a B ultrasound scoring system and exploring its application in the clinical diagnosis and treatment of pernicious placenta previa (PPP). 60 patients with PPP were divided into a low-risk group (severe, implantable) and high-risk group (adhesive, penetrating) according to their clinical characteristics, B ultrasound imaging characteristics, and postpartum pathological examination results. Under PPP ultrasonic image information using the deep learning algorithm, the B ultrasound image diagnostic scoring system was established to predict the depth of various types of placenta accreta. The results showed that the cut-off values of severe, implantable, adhesive, and penetrating types were <2.3, 2.3-6.5, 6.5-9, and ≥9 points, respectively; there were significant differences in the termination of pregnancy and neonatal birth weight between the two groups (*P* < 0.05); the positive predictive value, negative predictive value, and false positive rate of ultrasound images based on the deep dictionary learning algorithm for PPP were 95.33%, 94.89%, and 3.56%, respectively. Thus, the ultrasound image diagnostic scoring system based on the deep learning algorithm has an important predictive role for PPP, which can provide a more targeted diagnosis and treatment plan for patients in clinical practice and improve the prediction and treatment efficiency.

## 1. Introduction

Pernicious placenta previa (PPP) is one of the critical obstetric diseases, which often causes uncontrollable massive hemorrhage in parturients, resulting in resection of the uterus, damage to surrounding organs, and even maternal death as well as adverse maternal and fetal outcomes such as iatrogenic preterm delivery and asphyxia in newborns [1, 2]. History of previous cesarean section and placenta previa are the main risk factors for PPP with placenta accreta [4]. In recent years, with the opening of the “three-child policy” in China, pregnant women who have previously undergone cesarean section choose to have another pregnancy, resulting in a significant increase in the incidence of PPP, which will continue to rise [5]. In PPP patients with placenta accreta, the most common maternal complication is postpartum hemorrhage, intraoperative hemorrhage will exceed 3,000 mL in 90% of parturients, and hemorrhage greater than 10,000 mL is not uncommon, causing a series of serious complications if not effectively controlled, such as hemorrhagic shock, disseminated intravascular coagulation (DIC), multiple organ failure, loss of fertility due to hysterectomy, and even death in severe cases [6, 7]. Literature showed that the hysterectomy rate caused by placenta accreta accounts for 73.3% of the perinatal hysterectomy rate, and the maternal mortality rate is as high as 7%, and the main complications of newborns are iatrogenic preterm delivery, stillbirth, and asphyxia [8]. Therefore, it is an important clinical topic for obstetric medical staff to clarify the preoperative diagnosis, scientifically and objectively assess its dangerousness, predict the possible intraoperative conditions, and select a reasonable and effective treatment plan to reduce the maternal hysterectomy rate and mortality, reduce maternal and fetal complications, and improve maternal and fetal outcomes [9].

The article "Deep Learning Algorithm-Based Ultrasound Image Information in Diagnosis and Treatment of Pernicious Placenta Previa" was published in 2022. Journal: Comput Math Methods Med.

Prenatal diagnosis of PPP is easier to make by ultrasound and magnetic resonance imaging (MRI), but whether it is associated with placenta accreta has been the focus and difficulty of clinical diagnosis [10]. As a noninvasive and reproducible examination, ultrasound has become the primary examination method for prenatal diagnosis of PPP and placenta accreta [11]. In order to improve the prediction of the dangers of prenatal diagnosis of PPP, foreign scholars found that ultrasound has a high positive and negative predictive value for placenta accreta; domestic scholars proposed the concept of the ultrasound scoring system for placenta accreta and pointed out that an ultrasound scoring scale has certain clinical value in predicting the dangers of placenta accreta and the type of accreta and can predict the risk of intraoperative bleeding and hysterectomy [12, 13].

As one of the algorithms in the field of machine learning, deep learning is a deep neural network with multiple hidden layers [14]. Dictionary learning is mainly based on the dictionary and coefficient solution of matrix decomposition. Deep dictionary learning combines the advantages of deep learning and dictionary learning, constructs a deep structure through multilevel dictionary learning, and constitutes a deep dictionary learning model to learn sample data to obtain a dictionary [15]. The current application of deep learning techniques in medical ultrasound image analysis mainly involves three tasks: classification, detection, and segmentation of various anatomical structures such as the breast, prostate, liver, heart, and fetus. In addition, 3D ultrasound provides a direction for improving ultrasound imaging diagnosis in clinical practice. The image reconstruction is mainly through learning model training sample data to obtain the dictionary and using the dictionary obtained by model learning to represent the input image to complete the process of image reconstruction [16]. Therefore, ultrasound image processing based on the deep learning algorithm was used to diagnose patients with PPP. The aim was to explore the diagnostic value of an ultrasound score for the disease and provide some theoretical basis for prenatal diagnosis of PPP patients.

The article "Deep Learning Algorithm-Based Ultrasound Image Information in Diagnosis and Treatment of Pernicious Placenta Previa" was published in 2022. Journal: Comput Math Methods Med.

## 2. Materials and Methods

### 2.1. General Information

Sixty patients with PPP admitted to hospital from January 1, 2018, to October 31, 2018, were selected as the study subjects. The patients and their families understood the situation and signed the informed consent, and this study had been approved by the ethics committee of hospital.

Inclusion criteria were as follows: (1) patients with gestational age ≥ 28 weeks, (2) patients with PPP diagnosed by pathology, (3) patients with a history of cesarean section, (4) patients who cooperate with the examination, and (5) patients with complete clinical data.

Exclusion criteria were as follows: (1) patients with complications during pregnancy, such as gestational hypertension and gestational diabetes; (2) patients with blood system diseases or patients with coagulation dysfunction and immune dysfunction; (3) patients with mental illness; (4) patients with uterine fibroids; and (5) patients with severe heart, liver, and kidney dysfunction. The general data of the patients are detailed in Table 1.

### 2.2. Ultrasonic Examination

All patients were examined by using a Doppler ultrasound diagnostic instrument. Abdominal probe frequency was 2.5~6.0 MHz; maximum display depth was 240 mm; superficial probe frequency was 6.5~10.0 MHz; maximum display depth was 150 mm. The patients were taken in supine position, and the abdomen was routinely examined. The attachment position, thickness, internal echo of the placenta, and the relationship between the posterior placenta and the uterine muscle wall were emphatically observed. The thickness of the lower uterine muscle layer was measured, and the posterior wall of the bladder was scanned continuously and smoothly to observe the relationship between the posterior wall of the bladder and the anterior wall of the uterus. All operations were performed by professional ultrasound physicians, and the patients with diagnostic difficulties were examined by two physicians simultaneously. Then, the ultrasonic image information was processed by the deep dictionary learning algorithm.

The article "Deep Learning Algorithm-Based Ultrasound Image Information in Diagnosis and Treatment of Pernicious Placenta Previa" was published in 2022. Journal: Comput Math Methods Med.

### 2.3. Diagnostic Criteria

PPP diagnostic criteria: there was a history of cesarean section or myomectomy; the pregnancy was placenta previa, and the placenta was attached to the original surgical scar; the risks of placental adhesions, accreta, and fatal bleeding were high; the placenta (attached to the lower segment and lower edge of the uterus) reached or covered the cervix, below the exposed part of the fetus.

Diagnostic criteria for the adherent placenta [17] were described as follows. With the gold standard, postoperative histopathology report showed uterine smooth muscle placental villi. However, in clinical practice, histopathology was combined with clinical diagnosis due to the lack of histopathological specimens. Clinical diagnosis basis was as follows: after the fetus was born smoothly, the placenta could not be delivered for a long time. Inflammatory changes in the decidua or excessive growth of the leaf-like villi leads to abnormal placenta accreta; the villi penetrated deep into the basal layer of the decidua, and the placenta adhered to the uterine wall.

The diagnostic criteria for neonatal asphyxia were the ones proposed by the expert consensus on diagnosis of neonatal asphyxia of the Chinese Academy of Traditional Chinese Medicine in 2016 (Table 2).

### 2.4. Ultrasound Diagnostic Criteria and Medical History Assessment for Prenatal PPP

Based on the ultrasound scoring scale for placenta accreta, after a period of trial, the ultrasound diagnostic scoring scale was developed. The ultrasound scoring scale consists of 6 dimensions, each with 2 points and a full score of 12 points (Table 3). According to the research reports of scholars, with the increase in the number of cesarean sections, the incidence of placenta previa with placenta accreta increased. The score of placenta accreta history was developed as follows: (1) a history of cesarean section (score 1) and times of cesarean section greater than or equal to 2 times (score 2); (2) no prenatal bleeding symptoms (score 0); otherwise, score 2; and (3) a history of abortion or vaginal delivery (score 1) and times of abortion or vaginal delivery greater than or equal to 2 times (score 2) (Table 4).

### 2.5. Deep Dictionary Learning Algorithm

Both deep learning and dictionary learning represent learning fields. The difference between them is that deep learning is input-representation, and dictionary learning is representation-input. The Euclidean cost function of dictionary learning is shown in

(1) $$\begin{array}{c} \underset{C,S}{\min}{\left\|Y-C•S\right\|}_{F}^{2}. \end{array}$$

The goal of traditional single-layer dictionary is to decompose the input signal *Y* into dictionary *C* and coefficient *S* by matrix decomposition; namely, it is assumed that the sample data set *Y* = {*y*_1_, *y*_2_, ⋯, *y*_*n*_}; the goal of dictionary learning is to represent the input data *Y* as the product of *C* and *S* matrices.

(2) $$\begin{array}{c} Y=C•S. \end{array}$$

*C* = {*c*_1_, *c*_2_, ⋯, *c*_*k*_} refers to the dictionary. Each column of *C* represents one atom, and each atom is a normalized vector. *S* = {*s*_1_, *s*_2_, ⋯, *s*_*n*_} corresponds to the coefficient matrix of sparse representation. The objective function of a dictionary learning optimization problem can be expressed as

(3) $$\begin{array}{c} \underset{C,S}{\min}{\left\|Y-C•S\right\|}_{F}^{2}+\lambda •{\left\|S\right\|}_{1}. \end{array}$$

*Y* is the training data set, *C* is the feature dictionary, and *S* is the corresponding coefficient matrix.

The article "Deep Learning Algorithm-Based Ultrasound Image Information in Diagnosis and Treatment of Pernicious Placenta Previa" was published in 2022. Journal: Comput Math Methods Med.

The mathematical representation of the deep dictionary learning model is shown in

(4) $$\begin{array}{c} Y=C_{1}•C_{2}\cdots •C_{n}•S_{i}. \end{array}$$

Multilayer dictionary learning, also known as multilayer matrix decomposition, adds the calculation amount of parameters and objective function, and the limited number of training data is easy to cause the overfitting problem. Therefore, in the process of multilayer dictionary learning, the deep dictionary learning model uses the training mode similar to SAE and DBN models. Hierarchical training ensures the convergence of each layer training and prevents overfitting. Its objective function is shown in

(5) $$\begin{array}{c} \underset{C_{r},S}{\min}{\left\|Y-C_{r}•S\right\|}_{F}^{2}+\lambda •{\left\|S\right\|}_{1},C_{r}=C_{1}C_{2}\cdots C_{n}. \end{array}$$

*C*_1_ *C*_2_ ⋯ *C*_*n*_ represents the dictionary trained for each layer of data.

For the *n*-layer deep dictionary learning model, the representation of the first-layer dictionary satisfies the following conditions.

(6) $$\begin{array}{c} \underset{S}{\min}{\left\|Y-C_{1}S_{1}\right\|}_{F}^{2}⟶S_{1},\\ \underset{C}{\min}{\left\|Y-C_{1}S_{1}\right\|}_{F}^{2}⟶C_{1}. \end{array}$$

The representation of intermediate dictionary satisfies the following conditions.

(7) $$\begin{array}{c} \underset{S_{i}}{\min}{\left\|S_{i-1}-C_{i}S_{i}\right\|}_{F}^{2}⟶S_{i},\\ \underset{C_{i}}{\min}{\left\|S_{i-1}-C_{i}S_{i}\right\|}_{F}^{2}⟶C_{i}. \end{array}$$

The representation of the last layer dictionary satisfies the following conditions.

(8) $$\begin{array}{c} \underset{S_{n}}{\min}{\left\|S_{n-1}-C_{n}S_{n}\right\|}_{F}^{2}⟶S_{n},\\ \underset{C_{n}}{\min}{\left\|S_{n-1}-C_{n}S_{n}\right\|}_{F}^{2}⟶C_{n}. \end{array}$$

Due to the use of linear decomposition in the training process, the final dictionary *C* of deep dictionary learning for *n*-layer can be represented as

(9) $$\begin{array}{c} C=C_{1}•C_{2}\cdots •C_{n}. \end{array}$$

The process of deep dictionary training includes three parts: data preprocessing, dictionary initialization, and dictionary updating.

The article "Deep Learning Algorithm-Based Ultrasound Image Information in Diagnosis and Treatment of Pernicious Placenta Previa" was published in 2022. Journal: Comput Math Methods Med.

Data preprocessing: the training samples need to be decomposed into image blocks, and the natural image requires grayscale processing of the sample image, and then, the gray image is decomposed into 8 × 8 image blocks.

Dictionary initialization: the dictionary is usually initialized by random initialization, but this can lead to variable results. QR decomposition with the advantages of stability has great differences among the samples obtained after decomposition. However, when the QR decomposition algorithm initializes the dictionary, the dimension of the dictionary is affected by the size of the training sample data. When the data sample is small, the generated dictionary dimension feature is too small to contain all the sample features. Therefore, the first *n* columns of the sample data are selected as initialized dictionary *C*_1_. The input of the second layer is the output coefficient matrix of the first layer. The dictionary is initialized layer by layer, and the initial dictionary is the *m* × *n* matrix. The equation for solving the initial coefficient is shown as follows.

(10) $$\begin{array}{c} S=C^{-1}•Y. \end{array}$$

*C* is the initial dictionary matrix, *S* is the expected initial coefficient matrix, and *Y* is the sample data. By calculating the inverse matrix of the dictionary and the inner product of the input data, the coefficient matrix is obtained.

Dictionary update: the dictionary is also updated layer by layer, and equation (11) is used to update the dictionary.

(11) $$\begin{array}{c} C=Y•S^{-1}. \end{array}$$

The dictionary is updated by solving the inverse matrix of the coefficient matrix and the inner product of the input sample.

Coefficient update: step 1: line merging of the input data of the current layer with the product of the next layer and coefficient of the dictionary is performed to get the matrix *Y*_*i*_; step 2: on the basis of updating the end dictionary in each layer, a unit diagonal matrix of the same size is merged in the row to get the matrix *B*_*i*_; step 3: using equation (10), the least square solution of the coefficient matrix *S*_*i*_ is obtained, which is related to the matrix *B*_*i*_ and *Y*_*i*_. In the iteration number of the algorithm, the dictionaries and coefficients of each layer are updated in the above. In the dictionary learning process of each layer, dictionary *C* and coefficient *S* should meet the following conditions.

(12) $$\begin{array}{c} \underset{S}{\min}{\left\|Y-C_{n-1}S\right\|}_{F}^{2}⟶S_{n},\\ \underset{C}{\min}{\left\|Y-{CS}_{n}\right\|}_{F}^{2}⟶C_{n}. \end{array}$$

The above two equations are least squares problems with closed solutions. In the learning process of each layer, the dictionary and coefficient are updated in the form of alternating minimization; that is, the *C* is fixed to optimize *S*, and then, the *S* is fixed to optimize *C*. Alternately updating the dictionary and coefficient will continue until the algorithm converges to a local minimum. *S*_*n*_ and *C*_*n*_ represent the coefficient matrix and dictionary learned at layer *n*, respectively.

The article "Deep Learning Algorithm-Based Ultrasound Image Information in Diagnosis and Treatment of Pernicious Placenta Previa" was published in 2022. Journal: Comput Math Methods Med.

### 2.6. Statistical Analysis

All the data were analyzed by SPSS 22.0. Measurement data of normal distribution were expressed as mean ± standard deviation ($\bar{x}\pm s$); the *t*-test was used; the measurement data of nonnormal distribution were represented by *M* (*Q*), and the *t*-test was adopted. Count data was expressed as *n* (%), using the *χ*^2^ test or Fisher's exact test. The receiver operating characteristic (ROC) curve was drawn, the area under the curve (AUC) was calculated, and the comprehensive score cut-off value of each type of placenta accreta was calculated. When *P* < 0.05, the difference was statistically significant.

## 3. Results

### 3.1. Patient Grouping

According to the ultrasound scoring scale and comprehensive score table of medical history, there are a total of 18 points. The mean score of the 60 patients was 2-14 points, with a mean of 7.8 ± 2.4 points. The ROC curve was used to obtain cut-off values for various types of placenta accreta. Patients were grouped according to cut-off values.

1. Low-risk group of placenta accreta: 27 patients with <6.5 points were given routine cesarean section to terminate pregnancy. According to the score, the patients could be divided into two groups: <2.3 points group, 10 cases in total, which were considered severe placenta previa, and 2.3-6.5 points group, 17 cases in total, which were considered implantable placenta previa
2. High-risk group of placenta accreta: a total of 33 patients with ≥6.5 points underwent ultrasound-guided temporary occlusion of the abdominal aorta balloon to terminate pregnancy. According to the score, the patients could be further divided into the ≥9 points group, with a total of 21 cases, which were considered to be penetrating placenta previa, and the 6.5-9 points group, with a total of 12 cases, which were considered to be adhesive placenta previa

60 patients with PPP can be divided into four groups: severe, implantable, adhesive, and penetrating. The ultrasound images and histopathological images before and after processing by the deep dictionary learning algorithm are shown in Figures 1 and 2.

The article "Deep Learning Algorithm-Based Ultrasound Image Information in Diagnosis and Treatment of Pernicious Placenta Previa" was published in 2022. Journal: Comput Math Methods Med.

### 3.2. Cut-off Value of Ultrasound Scoring Combined with Medical History in Predicting Various Types of Placenta Accreta

1. Severe and implanted types

AUC of ROC was 93.1%. The maximum AUC score of the Youden index (YI) was 2.1, the sensitivity was 82.9%, and the specificity was 86.6%. Therefore, the cut-off value for severe and implantable placenta previa was 2.3. Score < 2.3 was considered to indicate severe placenta previa, and score ≥ 2.3 was considered to indicate implantable placenta previa (Figure 3(a)).

(2) Implanted and adhesive types

AUC of the ROC curve was 93.4%, the maximum AUC score of YI was 6.3, the sensitivity was 77.8%, and the specificity was 85.5%. Therefore, the cut-off value of implantable and adhesive placenta previa was 6.5. Score < 6.5 was considered to indicate implantable placenta previa, and score ≥ 6.5 was considered to indicate adhesive placenta previa (Figure 3(b)).

(3) Adhesive and penetrating types

AUC of the ROC curve was 93.6%, the maximum AUC score of YI was 8.7, the sensitivity was 90.4%, and the specificity was 82.7%. Therefore, the cut-off value of adhesive and penetrating placenta previa was 9. Score < 9 was considered to indicate adhesive placenta previa, and score ≥ 9 was considered to indicate penetrating placenta previa (Figure 3(c)).

### 3.3. Comparison of Case Data between the Low-Risk Group and High-Risk Group

There was no significant difference in age, number of pregnancies, number of cesarean sections, number of abortions/vaginal deliveries, and preoperative hemoglobin (HGB) between the low-risk group and the high-risk group (*P* > 0.05). In terms of gestational age, the gestational age of termination of pregnancy in the high-risk group was 35.5 ± 0.7 weeks, which was earlier than that in the low-risk group (37.8 ± 0.6 weeks), and the difference was statistically significant (*P* < 0.05) (Figures 4 and 5).

### 3.4. Comparison of Maternal and Infant Conditions during Operation between the Low-Risk Group and High-Risk Group

There was no significant difference in operation time, intraoperative blood loss, and neonatal Apgar score between the low-risk group and the high-risk group (*P* > 0.05); the neonatal birth weight in the high-risk group was 3.7 ± 0.3 kg, which was significantly lower than that in the low-risk group (4.1 ± 0.1 kg) (*P* < 0.05), and the difference was statistically significant (Figures 6 and 7).

### 3.5. Comparison of Postoperative Condition between the Low-Risk Group and High-Risk Group

The patients in the low-risk group and high-risk group had stable vital signs, no ICU metastasis, and no related complications, and there was no significant difference between the two groups in postoperative hospital stay (*P* > 0.05) (Figure 8).

The article "Deep Learning Algorithm-Based Ultrasound Image Information in Diagnosis and Treatment of Pernicious Placenta Previa" was published in 2022. Journal: Comput Math Methods Med.

### 3.6. Ultrasonic Diagnosis Results

The positive predictive value, negative predictive value, and false positive rate of the ultrasound image information based on the deep dictionary learning algorithm for the PPP were 95.33%, 94.89%, and 3.56%, respectively (Figure 9).

## 4. Discussion

Because the specificity of medical images of PPP varies greatly, overdiagnosis or missed diagnosis sometimes occurs in clinical practice [18]. In recent years, it has been reported that the sensitivity, specificity, and positive predictive value of ultrasound in the diagnosis of PPP are 87%-95%, 76%-98%, and 82%-93%, respectively [19]. Ultrasound scoring combined with medical history was used for prenatal diagnosis of PPP and placenta accreta, and in 60 patients with PPP, 10, 17, 12, and 21 patients had severe, implantable, adhesive, and penetrating PPP, respectively. The positive predictive value, negative predictive value, and false positive rate of ultrasound image information based on the deep dictionary learning algorithm for PPP were 95.33%, 94.89%, and 3.56%, respectively. It is similar to the findings of Mosconi et al. [20]. Therefore, it is concluded that ultrasound scoring based on the deep dictionary learning algorithm combined with medical history has a good diagnostic value for PPP.

The researchers developed the ultrasound scoring scale for placenta accreta and proposed that the ultrasound evaluation thresholds for the three types of placenta accreta were adhesive type < 3 points, implantable type ≥ 3 points, and penetrating type ≥ 10 points [21]. However, the cut-off values for severe, implantable, adhesive, and penetrating types were <2.3, 2.3-6.5, 6.5-9, and ≥9 points, respectively. Because a large area of the placenta in the third trimester of pregnancy is in the uterus and its lower segment and some of them are attached to the cervix, it is difficult to observe the integrity of cervical morphology. In ultrasonography, the placental image at the uterus and its lower segment is mainly assessed, and the abnormal cervical canal during the assessment is classified into the lower segment of the uterine body; in the past, the analysis only considered the history of the cesarean section. In this discussion, three aspects were considered: the number of cesarean sections, the number of miscarriage vaginal delivery, and preoperative HGB. The former two are the factors of PPP, and preoperative HGB is an important indicator for assessing prenatal bleeding, so there are some differences between them.

The article "Deep Learning Algorithm-Based Ultrasound Image Information in Diagnosis and Treatment of Pernicious Placenta Previa" was published in 2022. Journal: Comput Math Methods Med.

In clinical practice, PPP is mainly treated by cesarean section, and patients with placenta accreta use different hemostatic regimens according to the depth of implantation during surgery. In recent years, there have been many studies on the PPP operation, but there are few relevant reports on different implantation types [22]. Patients with <6.5 points were divided into a low-risk group for placenta accreta and given conventional cesarean section to terminate pregnancy; patients with ≥6.5 points were divided into a high-risk group for placenta accreta and given ultrasound-guided temporary occlusion of abdominal aortic balloon to terminate pregnancy. The differences in the operation time, intraoperative blood loss, neonatal Apgar score, and postoperative hospital stay between the two groups had no statistical significance (*P* > 0.05). Patients with low risk of placenta accreta can undergo conventional cesarean section without significant effect on the fetus, which can not only save medical resources and avoid the related risks caused by vascular intervention but also reduce the economic burden of patients.

## 5. Conclusion

The ultrasound image information of PPP was processed by the deep dictionary learning algorithm, and a B ultrasound scoring system was constructed to explore its application value in the clinical diagnosis and treatment of the disease. It indicates that the ultrasound images under this algorithm have a high positive predictive value and negative predictive value for PPP; the B ultrasound image diagnostic scoring system can effectively obtain the cut-off value of severe, implantable, adhesive, and penetrating placenta accreta. The ultrasound image diagnostic scoring system based on the deep learning algorithm plays an important role in predicting PPP and can provide more targeted diagnosis and treatment plan for patients in clinical practice and improve the prediction and treatment efficiency. However, the sample size is relatively small, and the time is short. In the future, more case data need to be collected for comprehensive analysis, so as to obtain a more accurate diagnosis.

## Figures and Tables

**Figure 1:** Ultrasound images before and after processing by the deep dictionary learning algorithm: (a–d) the ultrasound images before processing by the deep dictionary learning algorithm; (e–h) the ultrasound images after processing by the deep dictionary learning algorithm; (a, e) the patient with severe placenta previa; (b, f) the patient with adhesive placenta previa; (c, g) the patient with implantable placenta previa; (d, h) the patient with penetrating placenta previa.

The article "Deep Learning Algorithm-Based Ultrasound Image Information in Diagnosis and Treatment of Pernicious Placenta Previa" was published in 2022. Journal: Comput Math Methods Med.

**Figure 2:** Histopathologic images of patients: (a–d) adhesive, implantable, implantable, and penetrating placenta previa, respectively (×200). The patients were 32, 28, 41, and 36 years old, respectively.

**Figure 3:** Ultrasound scoring combined with medical history to predict the cut-off value of various types of placenta accreta: (a) the cut-off value for severe and implantable placenta accreta; (b) the cut-off value for implantable and adhesive placenta accreta; (c) the cut-off value for adhesive and penetrating placenta accreta.

**Figure 4:** Comparison of age, gestational age, and preoperative HGB between the two groups. ∗ indicates that the difference was statistically significant (*P* < 0.05).

**Figure 5:** Comparison of pregnancy times, cesarean section times, and abortion/vaginal delivery times between the two groups.

**Figure 6:** Comparison of operation time, intraoperative blood loss, and neonatal birth weight between the two groups. ∗ indicates that the difference was statistically significant (*P* < 0.05).

**Figure 7:** Comparison of the neonatal Apgar score between the two groups.

**Figure 8:** Comparison of postoperative hospital stay between the two groups.

**Figure 9:** Ultrasonic diagnosis results.

**Table 1:** General data of the patients.

Age	Gestational age	Gravidity	Parity	Cesarean section history	Medication history

24-45 years	28-38 weeks	2-4 times	1-3 times	1-2 times	1-2 times
Average age	Average gestational age	Average gravidity	Average parity	Average cesarean section history	Average medication history
30.40 ± 2.32 years	34.41 ± 2.64 weeks	3.41 ± 0.63 times	2.41 ± 0.42 times	1.34 ± 0.22 times	1.24 ± 0.15 times

**Table 2:** Diagnostic criteria for neonatal asphyxia.

Conditions	Evaluation results	Specific performance
Blood gas analysis results	Mild asphyxia	Apgar score 1 min ≤ 7 points or 5 min ≤ 7 points, cord blood pH < 7.2
	Severe asphyxia	Apgar score 1 min ≤ 3 points or 5 min ≤ 5 points, cord blood pH < 7.0
No blood gas analysis results	Low Apgar score	Abnormal Apgar score
	Mild asphyxia	Apgar score 1 min ≤ 7 points
	Severe asphyxia	Apgar score 1 min ≤ 3 points

**Table 3:** Ultrasonic diagnostic scoring of placenta accreta.

	Placenta position	Placental thickness	Retroplacental space	Serosa of the urinary bladder	Placental sinus	Blood flow signal at the base of the placenta
0	Normal	<3 cm	Continuity	Continuity	None	Regular blood flow
1 point	Marginal or low-lying placenta (placenta 2 cm from the cervix)	3-5 cm	Local interrupt	Local interrupt	There is placental sinus	Increased blood flow into clusters
2 points	Complete placenta previa	>5 cm	Disappear	Disappear	Fusion into pieces, with “boiling water sign”	“Cross-border vessels” appear

The article "Deep Learning Algorithm-Based Ultrasound Image Information in Diagnosis and Treatment of Pernicious Placenta Previa" was published in 2022. Journal: Comput Math Methods Med.

**Table 4:** Placenta accreta history score scale.

History of cesarean section	Prenatal bleeding symptoms	History of abortion or vaginal delivery
Once, score 1	No, score 0	Once, score 1
≥2 times, score 2	Yes, score 2	≥2 times, score 2

## Data Availability

The data used to support the findings of this study are available from the corresponding author upon request.
